# New Construction of Family of MLCS Algorithms

**DOI:** 10.1155/2021/6636710

**Published:** 2021-01-19

**Authors:** Haihe Shi, Jun Wang

**Affiliations:** School of Computer and Information Engineering, Jiangxi Normal University, Nanchang, China

## Abstract

The multiple longest common subsequence (MLCS) problem involves finding all the longest common subsequences of multiple character sequences. This problem is encountered in a variety of areas, including data mining, text processing, and bioinformatics, and is particularly important for biological sequence analysis. By taking the MLCS problem and algorithms for its solution as research domain, this study analyzes the domain of multiple longest common subsequence algorithms, extracts features that algorithms in the domain do and do not have in common, and creates a domain feature model for the MLCS problem by using generic programming, domain engineering, abstraction, and related technologies. A component library for the domain is designed based on the feature model for the MLCS problem, and the partition and recur (PAR) platform is used to ensure that highly reliable MLCS algorithms can be quickly assembled through component assembly. This study provides a valuable reference for obtaining rapid solutions to problems of biological sequence analysis and improves the reliability and assembly flexibility of assembling algorithms.

## 1. Introduction

The problem of finding the longest common subsequence between sequences is called the *longest common subsequence* (LCS) problem, and that of finding the longest common subsequence among more than two sequences is called the *multiple longest common subsequence* (MLCS) problem. The MLCS problem was shown to be an NP-hard problem in [1]. This problem is widely used in the fields of bioinformatics and computational genomics [2–4]. The rapid development of high-throughput sequencing technology [5] has promoted the implementation of many international genomic projects [6], and massive amounts of data have been generated in the field of bioinformatics. This has led to the formation of large-scale bioinformatics data, where this scale continues to grow. The LCS of a set of biological sequences usually preserves informative segments (subsequences) that are conserved during the evolutionary process on the condition that no internal deletions or insertions occur within contiguous segments. Finding the LCS of biological sequences is the basic means and method of studying biological sequence data and forms the basis for further sequence analysis (such as multiple sequences alignment, gene prediction based on similarity, genome rearrangement, and so on).

For over 40 years, significant efforts have been made to find efficient algorithms for the MLCS problem. For the LCS problem, the most effective algorithm is the dynamic programming algorithm. The normal dynamic programming algorithm was first proposed by Wagner and Fischer in 1974 [7]. However, when searching the LCS of large-scale data, the normal dynamic programming algorithm has problems such as excessive memory space occupation and high time complexity. Therefore, the dynamic programming algorithms that optimize space complexity were proposed, such as Hirschberg algorithms [8], SB algorithms [9], and Smith-Waterman algorithms [10]. The dynamic programming algorithms can effectively solve the LCS problem of double sequences, but in practical applications, it is often necessary to deal with the MLCS problem of multiple sequences. As the number of sequences increases, the time and space complexity of the dynamic programming algorithms increase exponentially, resulting in a poor performance of the dynamic programming algorithms when dealing with MLCS problems. In order to solve this problem, many other MLCS algorithms have been proposed, which can be divided into the heuristic MLCS algorithms and the dominant point-based MLCS algorithms. The heuristic MLCS algorithms are approximate algorithms, and the dominant point-based MLCS algorithms are precise algorithms. The approximate algorithms for MLCS problem were first proposed in 1994 [11, 12], and then the Expa algorithm was successively proposed [13], as well as *best next for maximal available symbols* (BNMAS) algorithm [14, 15], *ant colony optimization* (ACO) algorithm [16], *beam search* (BS) algorithm [17], and so on. In the ACO algorithm, Shyu and Tsai transformed the MLCS search problem into a node state change problem in the ant colony algorithm and defined state transition rules and pheromone update rules. In the BS algorithm, Blum transforms the MLCS problem into a problem of tree search, first builds a search tree for all input sequences, and then uses the heuristic tree search algorithm, Beam search, to search for MLCS. The efficiency and solution quality of ACO algorithm and BS algorithm are better than other heuristic MLCS algorithms. In practical applications of MLCS problem, there are many cases where the exact solution needs to be calculated. Therefore, the dominant point-based algorithms are most widely used in the MLCS problem. In 1977, Hunt and Szymanski found that, when using dynamic programming algorithms to solve LCS problems [18], the actual data used is only the value of the position of a few points with the same characters in the dynamic programming score matrix, and the data at other positions in the score matrix can be deleted. According to the above findings, the idea of dominant point-based algorithm is proposed: by calculating the dominant points between a set of molecular sequences, and generating all the dominant point data into a *directed acyclic graph* (DAG), each longest path in the DAG is a longest common subsequence of the input sequences. Compared with the dynamic programming algorithm, it greatly reduces the time and space complexity. In 2006, Chen proposed the Fast_LCS algorithm first using the successor table (a data structure) [19]. The successor table can quickly calculate the match points of the molecular sequence and then quickly delete the redundant match points through a defined series of pruning operations to generate dominant points, thereby greatly reducing the time to generate a DAG. In 2011, wang proposed Quick_DP algorithm and its parallel algorithm Quick_DPPAR by improving the pruning function of Fast_LCS [20]. In 2016, Li proposed Top_MLCS algorithm [21] by constructing *Irredundant Common Subsequence Graph* (ICSG). ICSG removed all redundant and duplicate matching points, which greatly improved the efficiency of searching MLCS. In addition, there are some algorithms that use heuristic functions as pruning functions to delete redundant matching points, and achieve good results, such as ProMLCS algorithm [22], MLCS-A∗ algorithm [23], MLCS-APP algorithm [24], and so on.

Current research on the MLCS problem has focused on optimizing specific steps of particular algorithms [25] or their parallel implementation [26]. Due to the diversity and structural complexity of MLCS algorithms, many users cannot select appropriate algorithms that conform to the characteristics of the given sequence, where this may lead to unnecessary errors in the application process. Therefore, it is important to research MLCS algorithms at the level of domain abstraction. This paper uses generic programming [27], domain engineering, feature modeling [28–30], abstraction, and related technologies to study the MLCS problem. We consider MLCS algorithms as research domain and conduct a domain analysis. The *feature-oriented domain analysis* (FODA) [28] method is first used to establish the model for the MLCS domain. Following this, the PAR platform is used to describe, design, and implement components of the domain that are involved in the MLCS domain model to generate a highly abstract MLCS algorithms domain component library. Finally, this component library is used to assemble and generate executable MLCS algorithms.

## 2. Related Technology

### 2.1. Partition and Recur Method

*Partition and recur method* (PAR method) is a formal development method based on division and recursion [31–35]; it is a unified algorithm design method, covering a variety of known algorithm design techniques, including dynamic programming method, greedy method, divide and conquer method, exhaustive method, and so on. It contains an algorithm design language (Radl, recurrence-based algorithm design language), an *abstract generic programming language* (Apla), and a unified algorithm design and proof method, as well as a series of generation systems (the PAR platform). Among them, PAR provides formal support for the process of designing the Radl algorithm based on the problem; it provides automated support for the generation of the Radl algorithm from the Apla program to the executable language program.

PAR has established two formal program development paths, and its platform architecture is shown in Figure 1. The first is that, for the quantization problem, the PAR method can convert the Structured Natural Language (SNL) demand model into a Radl protocol model, and then into a Radl algorithm model, and then further into an Apla abstract program model, and finally into a high-level language program that can be run directly. The second way is, for non-quantitative problems, you can directly design the Apla program through the SNL demand model, supplemented by the corresponding formal proof, and then convert the Apla program into an executable program.

### 2.2. Domain Modeling

Software reuse is considered an effective means of solving the software crisis and implement the mode of industrialized production to the software industry [36]. Software reuse activity consists of two related phases: the production phase of reusable software assets, and the development phase of application systems based on reusable software assets [37]. Domain engineering corresponds to the stage of production of reusable software assets (system identification) and can develop and organize reusable software assets in the domain to provide the necessary material and technical foundation for the subsequent development of the application system.

Domain engineering is the main technical means of the production of reusable software assets. It consists of three stages: domain analysis, domain design, and domain realization. Domain analysis is based on an analysis of the requirements of several typical systems in the domain. It first considers such factors as expected changes in demand, technological development, and objective constraints to determine the appropriate scope of the domain. It then identifies the commonality and variability in the domain to obtain a set of domain requirements with sufficient reusability. Finally, it abstracts the requirements to form a domain model. Domain design and implementation is based on the domain model to identify, develop, and organize reusable assets, such as frameworks and components in the domain. When developing a new algorithm in the same field, we need to determine the requirements of the algorithm based on the domain model, select the appropriate algorithmic framework, and use this as the basis for selecting components for assembly to finally form the new algorithm. In this way, new algorithms are no longer developed from scratch but are based on the massive reuse of algorithmic components in the stages of analysis, design, and implementation.

FODA method [28] was introduced into the research and practice of domain engineering in 1990. FODA uses the relationship between features (feature model) as an important part of the domain model. Features in domain engineering can be divided into two categories: mandatory and variable features. Mandatory features are those that exist in all parts of the domain, and variable features are those that exist only in parts of the domain. Mandatory features clarify the commonality of the domain and variable features clarify its variability. Compared with commonality, variability is more important to study. Variable features can be divided into the following types:

1. Optional feature (optional), which represents an optional feature of the instance in the domain
2. XOR feature, which represents that the instance in the domain has and can only be selected one feature in a set of XOR features, because the XOR features are mutually exclusive
3. OR feature, which means that the instance in the domain contains at least one feature in a set of OR features

The mandatory feature and three variable features are represented in the domain model as shown in Figure 2. In this paper, the feature modeling method is used to establish the domain feature model for the domain of MLCS algorithms, and the abstract programming language Apla of the PAR platform is used to formally implement the component library of the domain.

### 2.3. Dominant Point

We use point *P*=[*p*_1_, *p*_2_,…, *p*_*n*_] to denote a unit in the dynamic programming scoring matrix *L* of *n* sequence, where *p*_*i*_(*i* ≤ *n*) represents the position of a character of sequence *a*_*i*_, and the value of position *P* in matrix *L* is *L*[*P*].

**Definition 1 .**

The point *P* is called the match point, if *a*_1_[*p*_1_]=*a*_2_[*p*_2_]=⋯=*a*_*n*_[*p*_*n*_]. That is, the characters of each sequence are consistent at point *P*.

**Definition 2 .**

For points *P*=[*p*_1_, *p*_2_,…, *p*_*n*_] and *Q*=[*q*_1_, *q*_2_,…, *q*_*n*_], if there is *p*_*j*_ ≤ *q*_*j*_ for all *j*(1 ≤ *j* ≤ *n*), then we call *P* dominating *Q*; if there is *p*_*j*_ < *q*_*j*_ for all *j*(1 ≤ *j* ≤ *n*), then we call *P* strong dominating *Q*.

**Definition 3 .**

Point *P* is a *k*-dominant point when the following conditions are true:

1. Point *P* is a match point
2. *L*[*P*]=*k*
3. There is no point *Q*(*Q* ≠ *P*), the value in the matrix *L* is *L*[*Q*]=*k*, and *Q* dominates *P*

## 3. MLCS Domain Modeling

### 3.1. Domain Analysis Process

This section invokes research on the commonly used MLCS algorithm and analyzes the domain of such algorithms. The FODA feature modeling method is used to perform feature modeling on the *service* (S), *function* (F), and *behavior characteristics* (B) in the domain of MLCS algorithm. The longest common subsequence search service is the core service in the field of MLCS. The main functions in this domain include *dynamic programming* (dp) algorithm operation, *heuristic multiple longest common subsequence* (HMLCS) algorithm operation, and the *dominant point-based multiple longest common subsequence* (DP-MLCS) operation. Among the core service, the dp algorithm operation and the HMLCS operation are optional functions, and the DP-MLCS algorithms operation is a mandatory function. The description of optional functions only focuses on its main components. For the mandatory function DP-MLCS, the main flow of its algorithm operation is described in detail. The dynamic programming mode selection (dp_mode) is a significant behavioral characteristic of the operation of the dynamic programming algorithm, including two main behavioral characteristics: *standard dynamic programming algorithm* (normal) and *dynamic programming algorithm that optimizes memory consumption* (space_opti). *Heuristic mode selection* (heur_mode) is a significant behavior characteristic of HMLCS. Here, only ACO algorithm and BS algorithm are taken as its main behavior characteristics. The operation process of the mandatory function DP-MLCS is as follows:

1. Check the validity of the sequence. The input of the algorithm is DNA sequence, and protein sequence. Before the algorithm is executed, the sequence information needs to be checked for validity to determine whether the input sequence is biologically significant.
2. Establish a preprocessing matrix for the input sequence. The data structure (successor table) was first proposed in [19] for preprocessing input sequences. In the literature, the successor table has been used to implement the Fast-LCS algorithm. Using the successor table and its pruning operation significantly reduces the time and space needed to calculate the match point. Most of the existing MLCS algorithms based on the dominant point use the successor table to preprocess the input sequence.
3. Use different pruning functions and heuristic functions to filter the match points, remove redundant match points, and calculate the dominant points contained in the match point set.
4. Use the obtained set of dominant points to establish directed acyclic graph (DAG), and each longest path in the DAG is a path of MLCS.
5. Backtrack to obtain all the longest common subsequence characters through a depth-first search and output the results.

The flow chart of DP-MLCS algorithms is shown in Figure 3.

Through accurate analysis of a series of DP-MLCS algorithms, the *successor table* (Successor Table, ST) operation, the *domination point calculation mode* (domi_mode) selection operation, the DAG operation, and the *result output* (result_op) operation are subfunctions of the DP-MLCS algorithms operation. The sequence legality check operation is the basic operation of the MLCS algorithm and is not described in the model. *Calculate match point* (CMP) and *pruning mode* (prune_mode) selection are the two significant behavior characteristics of the domi_mode selection operation. There are two main behavior characteristics under the prune_mode: *prune function* (PF) and *heuristic function* (HF). *Backtrack* (BT) is used as the significant behavioral characteristics of the result_op operation. The MLCS domain model is shown in Figure 4.

### 3.2. Domain Design Process

#### 3.2.1. Component Design

The domain is designed according to the above domain model of MLCS algorithms. The constraints and dependencies between the features are designed and analyzed, and the dependency graph of the algorithm component is established. This section only introduces the component dependencies of a series of DP-MLCS algorithms in the MLCS algorithms as a simple example. The algorithm input in this domain is molecular sequence. Before the algorithm is executed, the sequence needs to be checked for legality. Combined with the introduction of the operation steps of the DP-MLCS algorithms in Section 3.1, the main component of this type of algorithm is the *sequence legality check component* (seq_check component), *successor table component* (successor_matrix_mani component), *dominant point mode selection component* (dominant_mode component), directed acyclic graph component (DAG component), *result output component* (result_op component), *matching point calculation* component (cal_match_point component), and *backtrack componen*t. The line with arrows indicates the dependency relationship of one component to another component, and the dependency relationship between components is shown in Figure 5.

#### 3.2.2. Components Implementation

According to the above domain feature model and component dependency relationships of MLCS algorithms, the PAR platform is used to formally implement the domain component library. The Radl language is first used to accurately describe the functional specifications of components of the MLCS field, which are then integrated according to the dependencies between them to form an ADT. Finally, the abstract programming language Apla is used to implement all ADTs. The specifications of the key components cal_match_point and prune_mode in the DP-MLCS algorithms are as follows:

  1 cal_match_point component
   | [ in successor matrix: set of successor table;
    *n*: integer; init point : array of integer;
   out match_point: array of integer;
    match _matrix: set of match_ point;
   aux seqs : array of character; ] |
   AQ: init _point[*n*] = [0, 0, 0,…, 0] ∧ *n* ≥ 2
   AR: ∀ match_point [*i*1, *i*2,…, *in*]: match_ point ∈ match _matrix: seqs [1] [*i*1] = seqs [2] [*i*2] = … = seqs[*n*][*i*_*n*_]

In the formal specification, *in*, *out*, and *aux* are three keywords defined by the PAR platform, which represent input, output, and auxiliary variables. The auxiliary variables do not need to appear in the program implementation. The *array*, *boolean*, *integer* are predefined types in the PAR platform. *AQ* represents the preconditions required by the component, and *AR* represents the postconditions of the component. The cal_match_point component implements the function to calculate the match points of input sequence by inputting the successor table and the initial match points. The *successor matrix* is the set of successor tables; *n* is the number of input sequences; *match_matrix* is the set of calculated match points; and the auxiliary variable *seqs* represents the input sequence, which stores all characters of the input sequence.

   2 prune_mode component
   | [ in *k*: integer; match_matrix: set of all match_ point that level = *k*;
    *P* [*p*1, *p*2,…, *pn*]: array of integer;
    *Q* [q1, q2,…, qn]: array of integer;
   out flag: boolean] |
   AQ: *k* ≥ 0∧*P*∈ match_matrix
   AR: flag = (∀Q : Q∈(match_matrix-P): ∃i: 0 < *i* ≤ *n*: *p*[*i*] < q[*i*])

The prune_mode component deletes the redundant points in the matching points through the pruning function, thereby calculating the dominant point of the sequence. In the specification, *k* is the rank of the input matching point (the position of the point in the longest common subsequence); *match_matrix* is the set of matching points with level *k*; *P* and *Q* are the matching points with input level *k*. The output *flag* is a Boolean value. If it is true, it indicates that the point *P* is the dominant point. Otherwise, the point *P* is a redundant point and should be deleted.

By using abstract data types and abstract processes that write programs directly, the Apla language can describe algorithmic problems abstractly. This makes it easy to verify its correctness and in turn ensures the reliability of the program. As the input language of the program generation system of the PAR platform, Apla can be quickly and easily converted into C++, Java, Python, and other programming languages and platforms.

According to the MLCS domain feature model established above, and by considering the dependencies between components as well as the relationships between data types and functions in the domain, we use Apla to define and implement MLCS algorithms components to form a domain component library. Owing to limitations of space, only the formal implementation of the DP-MLCS algorithm is given, and the specific implementation code is omitted.

  1 Seqs ADT
  define ADT Seqs (sometype elem);
   type Seqs = private;
   procedure read_seqs ();
    function seq_check(Seqs): boolean;
    procedure Generate_successor_matrix (Seqs;
     proc successor_matrix (char_num, seq_num:integer;
     proc memory_successor_of_matrix (sometype elemMatrix));
    procedure set_value (*i*: integer; *j*: integer; *k*: integer);
    function get_value (*i*: integer; *j*: integer; *k*: integer): integer;
   enddef

Considering that the functions performed by the *seq_check* component and the *successor_matrix_mani* component are all dependent on the input sequence, the ADT *Seqs* encapsulates these two components as well as their auxiliary components. Because the type of input data is temporarily uncertain, a type parameter *elem* is defined. The function *read_seqs* is used to obtain all the sequences to be searched in the input text file. The function *seq_check* is the realization of the function of the component *seq_check* and is used to check the legality of the input sequences.

The subroutine *Generate_successor_matrix* is the realization of the function to the *successor_matrix_mani* component. The generic subroutine successor_matrix in *Generate_Successor_matrix* dynamically provides memory for the successor matrix according to the input data and initializes the successor matrix. Of the input parameters, *char_num* is the character type in the input sequences, and *seq_num* is the number of input sequences. This generic subprogram supports the instantiation of different forms of successor tables required by different algorithms. The *memory_successor_of_matrix* subroutine is responsible for calculating and storing the successor matrix of the input sequence. The *get_value* and *set_value* subprograms, respectively, obtain and set the value in successor_matrix.

   2 MatchPoint ADT
   define ADT MatchPoint (sometype elem);
   type MatchPoint = private;
   function cal_match_point (sometype elemMatrix): sometype elemMatrix;
   function pruning_tech (sometype elem Matrix, a : array[integer]): boolean;
   function memory_dominant_point (b : array[integer]): sometype elemMatrix;
   enddef

The ADT *MatchPoint* encapsulates the *dominant_mode* component related to operations of the match points. The ADT contains three functions. The first is the cal_match_point function to calculate the matching point, where elemMatrix is a type parameter. The second is generic function pruning_tech that chooses different pruning techniques according to the input matrix. This is a Boolean function used to determine whether the matching points satisfy the condition to become the dominant point. The third function is memory_dominant_point, used to store information relevant to the hierarchically dominant point.

   3 DAG ADT
   define ADT DAG (sometype elem)
   type DAG = private;
   function Generat_graph (sometype elemMatrix): sometype elemMatrix;
   procedure backtrack (sometype elemMatrix; func print_MLCS(): string);
   enddef

The ADT *DAG* encapsulates three operational components related to directed acyclic graphs: the *DAG*, *backtrack*, and *result_op*. The function *Generat_graph* generates a DAG based on the set of the input dominant points, and the subprogram backtrack uses a depth-first search strategy to traverse the DAG. According to the matrix of dominant point, the subprogram will choose different traversal methods, and it also includes a subfunction *print_MLCS*, which is used to output the obtained MLCS, and record and output the number of MLCS.

## 4. Applications

### 4.1. DP-MLCS Algorithm Assembly Based on ADT

We use the ADT of MLCS algorithm component established in Section 3.2.2 to assemble and generate one MLCS algorithm. Part of the program is as follows:

  Program MLCS:
   const path_infile: string;/^∗^ file path of input sequence^∗^/
   const path_outfile: string; /^∗^ file path of output MLCS^∗^/
   var
   seqs: Array [String];/^∗^save the input sequence ^∗^/;
   char_num, seq_num: integer;
   /∗ successor matrix initialization, omit the matrix initialization code ∗/
   function successor_matrix (char_num, seq_num);
   var
   *i*, *j*: integer;
   begin
   foreach (*i*, *j*: 0 ≤ *i* ≤ char_num, 0 ≤ *j* ≤ *n*)
   …;
   end
   /∗instantiation of functional components used by DP_LCS ∗/
   ADT Fast_Seqs: new Seqs ();
   ADT match_point: new MatchPoint (successor_matrix);
   ADT dag: new DAG (Memory_dominant_point);
   /∗MLCS Searching manipulate procedure∗/
   procedure MLCS_search_mani (Check; Matrix; Cal_match_point; Pruning_tech;
   Memory_dominant_point; Graph; TB);
   var
   match_matrix, dominant_matrix:array[array[integer]]
   begin
   Fast_Seqs. read_seqs (path_infile);
   Fast_Seqs. seq_check (seqs);
   Fast_Seqs. Generate_successor_matrix (seqs);
   match_point.cal_match_point (successor_matrix);
   match_point.pruning_tech (match_matrix);
   match_point.memory_dominant_point(dominant_matrix);
   graph = dag. Generat_graph (dominant_matrix);
   dag. backtrack (graph, result_op(path_outfile));
   end

### 4.2. Results

By using the Apla-C++ program generation system of the PAR platform, we convert the Apla program of the assembly algorithm into C++ code. The generic programs and functions defined in Apla were converted into separate class member functions in C++ to reduce the coupling between components. In particular, the calling functions were converted into indicator functions in C++, and the generic parameter was converted into the pointer parameter to implement the polymorphism of the Apla program. After converting all ADT components to C++, the Apla code of the MLCS search operation was converted into a main function, and finally an algorithm program that can be run was generated by manually assembling the components.

We tested our assembly algorithm on the rice gene sequence of the GenBank database and compared the performance of our assembly algorithm with that of Clustal-W algorithm [38], which is a popular algorithm for multiple-sequence alignment and MLCS. First, we experimented with different numbers of DNA sequences when the sequence length is 50; the computation time of MLCS to the two algorithms is shown in Table 1. Second, we tested the two algorithms on five sequences sets with different lengths; the result is shown in Table 2, and one computation result of the assembly algorithm is shown in Figure 6. From Tables 1 and 2, we can see that our assembly algorithm is faster than Clustal-W for sets with different numbers of sequences and sequences sets with different lengths. Because Clustal-W is not an exclusive algorithm for MLCS problems, the accuracy rate of MLCS obtained by it is also lower than that of the DP-MLCS algorithm we assembled.

Because of the excellent verifiability of high-level language Apla, the MLCS algorithm formed by component assembly in the domain of MLCS not only improves the reliability, execution efficiency, and maintainability of the assembly algorithm program, but also can be manually assembled to form the specified algorithm according to customer needs, and also enhances the generality of algorithm components.

## 5. Conclusion

Sequence alignment is a key method and problem in research on bioinformatics. Finding the longest common subsequence among multiple biological sequences is an effective technique for sequence alignment. The MLCS algorithms are widely used in bioinformatics, data mining, information retrieval, and pattern recognition. This article is the first to consider algorithms to solve the MLCS problem as a special field, research them at a high level of abstraction, improve their reliability and developmental efficiency, and reduce the likelihood of occurrence of suboptimal solutions and errors. We used FODA method to analyze the domain of the MLCS algorithms, extract its general and variable features, and transform them into components. The formalized specification language Radl was used to accurately describe the functional specifications of components of MLCS algorithms, and the high-level language Apla was used to implement the function components. Automatic or semiautomatic methods are expected to be available to solve the problems of the assembly and generation of highly reliable components for specific problems. Finally, through a series of program conversion systems on the PAR platform, it is quickly converted into executable algorithms. The final experimental results show that our research has high practicability.

This paper combines the theories and techniques of domain engineering, generative programming, formal methods, etc., and the practical research carried out on the MLCS algorithm family can provide new ideas for algorithm research in other fields of bioinformatics. We have applied this research method to the study of pairwise sequence alignment problems and multiple-sequence alignment problems and have achieved substantial achievement. This shows that the algorithmic assembly generation method in this paper is extended to other types of problems and is expected to develop into a method to solve a series of similar problems. Next, we will design a graphical user interface (GUI) for the component library to enable users to obtain the required algorithms by selecting components on the visual interface.

## Figures and Tables

**Figure 1:** Platform architecture of PAR, it contains two formal program development paths.

**Figure 2:** Representation of four feature relationships. (a) Mandatory feature, (b) Optional feature, (c) XOR feature, and (d) OR feature.

**Figure 3:** Operation flow chart of DP-MLCS algorithms. Arrows indicate the sequence of operations.

**Figure 4:** Domain feature model of MLCS algorithms, boxes represent features, and lines with dots represent the relationship between features.

**Figure 5:** Dependency relationships of component to DP-MLCS. The line with arrows indicates the dependency relationship of one component to another component.

**Figure 6:** One experimental result of the assembly algorithm, which contains the input sequence, all MLCS, and the number and length of MLCS.

**Table 1:** Comparison of computation time of assembly algorithm and that of Clustal-W on sequences sets with different numbers of sequences.

Sequence number	Time of assembly algorithm (ms)	Time of Clustal-W (ms)
3	597	760
5	2046	2559
7	5885	6657
9	6970	8120

**Table 2:** Comparison of computation time of assembly algorithm and that of Clustal-W on sequences sets with different lengths.

Sequence length	Time of assembly algorithm (ms)	Time of Clustal-W (ms)
30	200	176
50	2145	2443
70	6878	7600
90	17654	21565
110	45568	60780

## Data Availability

The datasets generated for this study are available on request to the corresponding author.
